The article "The Oral Wound Healing Potential of Thai Propolis Based on Its Antioxidant Activity and Stimulation of Oral Fibroblast Migration and Proliferation" was published in 2022. Journal: Evid Based Complement Alternat Med.

# The Oral Wound Healing Potential of Thai Propolis Based on Its Antioxidant Activity and Stimulation of Oral Fibroblast Migration and Proliferation

**DOI:** 10.1155/2022/3503164

**Published:** 2022-05-26

**Authors:** Suppanut Jongjitaree, Sittichai Koontongkaew, Nattisa Niyomtham, Boon-ek Yingyongnarongkul, Kusumawadee Utispan

**Affiliations:** ^1^Faculty of Dentistry, Thammasat University, Bangkok, Thailand; ^2^Walailak University International College of Dentistry, Walailak University, Bangkok, Thailand; ^3^Department of Chemistry and Center of Excellence for Innovation in Chemistry (PERCH-CIC), Faculty of Science, Ramkhamhaeng University, Bangkok, Thailand

## Abstract

**Introduction:**

Propolis has demonstrated wound healing effects. Propolis' effects vary based on its composition and geographical origin. However, there are few reports on the effects of propolis on oral wound healing. The aim of this study was to evaluate the antioxidant and *in vitro* gingival wound healing effects of the *n*-hexane extract of propolis (HEP), ethyl acetate extract of propolis (EEP), and aqueous extract of propolis (AEP) fractions of the ethanol extract of Thai propolis.

**Materials and Methods:**

The crude ethanol extract of propolis was obtained by maceration with 95% ethanol that was sequentially fractionated with hexane, ethyl acetate, and distilled water. The chemical profiles of the samples were assessed by thin-layer chromatography (TLC) and gas chromatography-mass spectrometry (GC-MS). Antioxidant activity was determined using DPPH and FRAP assays. The effects of the propolis fractions on human gingival fibroblast (HGF) proliferation, migration, and *in vitro* wound healing were determined by MTT, modified Boyden chamber, and scratch assay, respectively.

**Results:**

We found that solvent polarity greatly affected the extract yield and TLC profiles. The highest extract yield was found in HEP (38.88%), followed by EEP (19.8%) and AEP (1.42%). TLC revealed 7 spots in the crude ethanol extract (Rf 0.36–0.80), 6 spots in HEP (Rf 0.42–0.80) and EEP (Rf 0.36–0.72), and 4 spots in AEP (Rf 0.17–0.79). GC-MS analysis revealed a high amount of triterpenoids in HEP (82.97%) compared with EEP (28.96%). However, no triterpenoid was found in AEP. The highest antioxidant activity and stimulation of HGF proliferation were observed in HEP, followed by EEP and AEP. HEP and EEP, but not AEP, enhanced HGF migration. However, all propolis fractions induced wound closure.

**Conclusions:**

HEP contained a large amount of triterpenoids. Antioxidant and *in vitro* wound closure effects were found in HEP, EEP, and AEP fractions.

## 1. Introduction

Oral wound healing is a complex process involving a cascade of well-orchestrated biological events that regulate the repair of oral tissue lesions. Healing consists of four phases, inflammation, proliferation, remodeling, and homeostasis. Although oral and dermal wound healing contain similar stages, oral wounds are characterized by rapid healing with minimal scar formation, mediated in part via an enhanced oral fibroblast and oral epithelial cell repair response [1].

Successful wound healing is accomplished by a series of coordinated processes that include cell migration and proliferation, extracellular matrix deposition, and remodeling. Fibroblasts are the most abundant cell type in connective tissue. These cells are involved in producing and remodeling the extracellular matrix [2]. Gingival fibroblasts play a critical role during oral wound healing and are required to regenerate connective tissue. These roles involve secreting matrix molecules and organizing these matrix components into functionally active fibers that restore the damaged oral tissues [3].

It has been demonstrated that oxygen is required to disinfect a wound; therefore, oxygen-dependent redox-sensitive signaling is an important process for regulating oxygen levels during the wound healing cascade. Formation of free radicals in tissues can directly impair the function of some aspects of the cell membrane or intracellular organelles or can initiate an inflammatory signaling pathway that leads to the production of numerous mediators of cell injury. The process of wound healing is largely impeded by excessive oxidative stress in a wound. The excessive reactive oxygen species (ROS) accumulated in the wound induce strong inflammatory reactions that can inhibit wound healing. Moreover, ROS inhibit the functions of endogenous stem cells and macrophages, slowing wound tissue regeneration [4, 5].

The interest in evidence-based complementary and alternative medicine has increased, resulting in many studies on the use of natural products for wound healing. Propolis, or bee glue, is a natural resinous substance collected by honeybees from tree buds and exudates. It consists mainly of resins, balsams, beeswax, essential oils, pollen, and other organic compounds. Propolis has antimicrobial, antioxidative, immunomodulatory, antiulcer, and wound healing effects. Therefore, it has been extensively used in the health industry worldwide [6, 7]. Propolis and its phenolic and flavonoid constituents have many therapeutic uses in oral health. A wide range of therapeutic uses due to its antibacterial, antiviral, antifungal, anti-inflammatory, wound and bone healing, and anticancer effects have been demonstrated in various *in vitro*, *in vivo*, and *ex vivo* studies, as well as in human clinical trials [8, 9].

The components of propolis vary. The characterization of the phenolic and flavonoid contents in propolis is needed to obtain the best therapeutic and medicinal benefits in dentistry and medicine [10]. Although many studies have been conducted to evaluate the healing effect of various therapeutic agents by focusing on skin wounds, few have evaluated oral wounds. Previous studies investigated the effects of Brazilian, Indian, Iranian, and Malaysian propolis on skin wound healing [11–13]. Solvent types and polarity impact the quality, quantity, and bioactivity of a natural product extract [14]. Furthermore, it was reported that the antioxidant capacity of propolis depended on the solvents used for extraction [15]. However, there is a lack of studies investigating the chemical profile and antioxidant activity based on the solvent extraction and the oral wound healing effect of Thai propolis. The aim of this study was to determine the phytochemical profile and the antioxidant activity of sequential hexane, ethyl acetate, and aqueous extracts of Thai propolis and to evaluate their oral wound healing effects on human gingival fibroblast proliferation and migration.

## 2. Materials and Methods

### 2.1. Chemicals

95% ethanol (analytical grade), methanol (analytical grade), ethyl acetate (analytical grade), and n-hexane (analytical grade) were purchased from Apex Alco Co., Ltd. (Bangkok, Thailand). Quercetin, gallic acid, galangin, naringenin, apigenin, *p-*anisaldehyde, dimethyl sulfoxide (DMSO), 1,1-diphenyl-2-picrylhydrazine (DPPH), and pyridine (HPLC grade) were purchased from Sigma-Aldrich (St. Louis, MO, USA). Dichloromethane (analytical grade) and formic acid were purchased from Thermo Fisher Scientific (Waltham, MA, USA). Bis(trimethylsilyl)trifluoroacetamide (BSTFA) with 1% trimethylchlorosilane (TMCS) was purchased from Cerilliant Corporation (Round Rock, TX, USA).

### 2.2. Propolis Extraction

Raw propolis (163 g) from *Tetragonula fuscobalteata* was harvested from an orchard in Chiang Mai province in Northern Thailand in January 2018 and kindly provided by Professor Somnuk Boongird, Faculty of Science, Ramkhamhaeng University. The preparation and extraction process was modified from Szliszka et al. [16]. Propolis (163 g) was divided into three equal parts (54.3 g each). Each aliquot of propolis (54.3 g) was dissolved in 150 mL of 95% ethanol and was shaken on an orbital shaker at 30 rpm in the dark. After 40 h, the macerated mixture was filtered using clean cotton wool and then a No.1 Whatman filter (Whatman, Marlborough, MA, USA). The procedure was repeated four times. The three propolis extract batches were combined and dried using a rotary evaporator (BUCHI R-300) (BUCHI Labortechnik AG, Switzerland) under reduced pressure at 60°C. The dried extracts were labeled as crude ethanol extracts and stored at −20°C.

### 2.3. Liquid-Liquid Partitioning

The partitioning process of crude propolis was modified from de Mendonca et al. [17]. The crude ethanol extract (98.04 g) was dissolved in 100 mL methanol to make the mother solution that was sequentially partitioned using three types of solvents (*n*-hexane, ethyl acetate, and water) in order of increasing polarity with a separating funnel. The methanol solution was partitioned with *n*-hexane (2 × 200 mL). The *n*-hexane layers were pooled and dried using a rotary evaporator. The methanol layers were pooled, dried, and dissolved with 100 mL of distilled water to obtain the aqueous-methanol extract. The aqueous-methanol extract was further partitioned with ethyl acetate (2 × 200 mL). The ethyl acetate and aqueous layers were collected separately. Each extract was pooled and dried using a rotatory evaporator. The dry weight of each partition was recorded as total yield. After separation, 63.37 g of the *n*-hexane extract of propolis (HEP), 32.34 g of the ethyl acetate extract of propolis (EEP), and 2.33 g of the aqueous extract of propolis (AEP) were obtained (Figure 1).

### 2.4. Qualitative Thin-Layer Chromatography

Thin-layer chromatographic (TLC) plates, composed of a 0.2 mm thick precoated silica gel 60F-254 layer (precoated TLC-sheets ALUGRAM Xtra SIL, G/UV 254 from Macherey-Nagel, Germany), received 1 *μ*L of the propolis extracts (containing 50–100 *μ*g of propolis extract), placed 1 cm from the lower edge of the plate. Preliminary TLC separation of the extracts was performed using different solvent systems; the solvent front was allowed to travel to at least 75% of the TLC plate height. Two solvent systems, *n*-hexane : ethyl acetate : formic acid (30 : 70 : 1) as a combination of nonpolar solvents and ethyl acetate : methanol : formic acid (50 : 50 : 1) as a combination of polar solvents, were used to elute the compounds in the extracts [18]. The spots were visualized using natural light, short wave ultraviolet (254 nm), and long wave ultraviolet (366 nm) for detecting the fluorescence compounds and by spraying with an anisaldehyde-sulfuric acid agent followed by heating at 110°C for detecting triterpenoids [19]. Finally, the TLC plates were photographed by a TLC visualizer 2 (CAMAG, Muttenz, Switzerland). Each spot was marked, and the retardation factor (Rf) value was calculated. The Rf value of the separated compound was defined as the distance travelled by the compound divided by the distance travelled by the solvent (the solvent front).

### 2.5. Gas Chromatography-Mass Spectrometry

The propolis extracts were derivatized prior to gas chromatography-mass spectrometry (GC-MS) analysis as previously described [20]. The dried propolis extract (30 mg) was dissolved in 1 mL pyridine mixed with BSTFA containing 1% TMCS solution (pyridine:1% TMCS BSTFA ratio 1 : 2). The solution was mixed in a sealed glass tube and incubated at 100°C for 30 min. The derivatized samples (1 *μ*L) were injected and analyzed by GC-MS.

The chemical compositions of the propolis extracts and standard compounds (*m-*coumaric acid, ferulic acid, caffeic acid, galangin, naringenin, apigenin, and quercetin) were characterized by GC-MS analysis. Each standard compound (2 mg/mL) was prepared in pyridine mixed with 1% TMCS BSTFA solution. An Agilent 7890 B/5977A Series Gas Chromatograph/Mass Selective Detector System with an autosampler model GC Sampler 80 (Agilent Technologies, Santa Clara, CA, USA) was used in this study. The MS was operated in the electron ionization mode (70 eV). Helium was employed as the carrier gas, and its flow rate was adjusted to 0.8 mL/min. The chromatographic separation of the chemical compositions was performed on a GC capillary column HP-5MS (30 m × 0.25 mm inner diameter and 0.25 *μ*m film thickness, Agilent Technologies). The initial temperature of the column was set at 60°C, then increased by 5°C /min to 300°C, and held for 10 min. The injector temperature was set at 320°C in the split mode (split ratio 10 : 1). The temperature of the GC-MS interface and ion source was set at 300°C and 230°C, respectively. The MS was operated in the full scan mode, and the MS scan range was 35–800 *m/z*. Interpretation of the GC-MS mass spectrum was performed using the Wiley Registry® 10th Edition/NIST 2014 Mass Spectral Library database. The mass spectrum of the unknown compounds was compared with the spectrum of specific standards and reference compounds in the library. An MS match score in the range of 70–100% was reported as the identified compounds in our propolis extracts [21]. The name, molecular weight, and molecular formula of the components of the test extracts were ascertained. The relative percentage amount of each compound was calculated by comparing its average peak area to the total peak area.

### 2.6. *In Vitro* Antioxidant Activity of Propolis Extracts

To evaluate the antioxidant activity of the propolis extracts, diphenylpicrylhydrazyl (DPPH) and ferric reducing antioxidant power (FRAP) assays were performed. Quercetin was used as a positive control in these assays.

#### 2.6.1. DPPH Radical Scavenging Activity Assay

The DPPH assay was employed to evaluate the stable free radical scavenging activity by modifying previous methods [22, 23]. Briefly, a DPPH solution (0.25 mg/mL ethanol) was prepared. Each propolis extract (10 mg/mL) was dissolved in DMSO. Each propolis extract or quercetin was diluted in DPPH to final concentrations of 500 *μ*g/mL and 10 *μ*g/mL, respectively. The mixture of DPPH and propolis extracts or quercetin was added to a 96-well plate (100 *μ*L/well). The plate was incubated at 25°C for 30 min in the dark, after which the absorbance was read at 512 nm using a spectral scanning multimode reader (Varioskan® Flash Type 3001) (Thermo Fisher Scientific, Waltham, MA, USA). DPPH in DMSO was used as control. The DPPH radical scavenging activity was calculated as follows:

(1) $$\begin{array}{c} \text{antiradical activity}\left(\%\right)=100\times \left[\frac{A-B}{A}\right], \end{array}$$

where A is the absorbance of DPPH in DMSO (control) and B is the absorbance of DPPH in a propolis sample or quercetin.

The experiment was performed in triplicate, and three independent experiments were performed.

#### 2.6.2. Ferric Reducing Antioxidant Power Assay

The FRAP of the propolis extracts was determined using a previously described method based on the reduction of ferric tripyridyltriazine complex to ferrous tripyridyltriazine [24]. Briefly, working FRAP reagent (300 mM acetate buffer at pH 3.6, 10 mM TPTZ (2,4,6-tripyridyl-s-triazine) in 40 mM HCl, and 20 mM FeCl_3_.6H_2_O at a ratio of 10 : 1 : 1) was freshly prepared. Working FRAP reagent (175 *μ*L) was added to 25 *μ*L propolis extracts or quercetin in each well of 96-well plates. The plate was incubated at 37°C for 4 min. The absorbance was read spectrophotometrically at 593 nm. The percentage of ferric radical scavenging activity was calculated as shown follows:

(2) $$\begin{array}{c} \text{ferric radical scavenging activity}\left(\%\right)=100\times \left[\frac{Abs593\text{ propolis extract}}{Abs593\text{ quercetin}}\right]. \end{array}$$

The experiment was performed in triplicate, and three independent experiments were performed.

### 2.7. Human Gingival Fibroblast Isolation and Culture

Human gingival fibroblasts (HGFs) were isolated from the explants of healthy gingival tissues from patients who underwent minor oral surgery at Thammasat University Hospital. The protocol for human tissue acquisition was performed according to the International Conference on Harmonization-Good Clinical Practice (ICH-GCP) and was approved by the Institutional Review Board of Thammasat University (IRB number 043/2562). The HGFs were isolated and cultured as previously described [25]. The HGFs were cultured in Dulbecco's Modified Eagle's Medium (DMEM) (Invitrogen, Carlsbad, CA, USA) containing 10% fetal bovine serum (FBS), 1% penicillin/streptomycin, and 1% amphotericin B. The HGFs were trypsinized when their confluence reached 80%. The 3rd–7th passage cells were used in the subsequent experiments.

### 2.8. Cell Proliferation Assay

HGFs were cultured in 96-well plates (3 × 10^3^ cells/well) for 24 h. The cells were treated with HEP (15.62, 31.25, 62.5, 125, or 250 *μ*g/mL), EEP (20, 40, 80, 160, or 320 *μ*g/mL), or AEP (200, 400, 600, 800, or 1000 *μ*g/mL) for 24 h. The cell proliferation in each treatment group was determined using the thiazolyl blue tetrazolium bromide (MTT) (Sigma) as previously reported [26]. The absorbance (Abs) of the solution was measured at 570 nm by a microplate reader (Tecan, Salzburg, Austria). The cell proliferation (%) relative to the control wells containing cell culture medium without test samples as a vehicle was calculated using [(A) test/(A) control] × 100, where (A) test is the absorbance of the test sample and (A) control is the absorbance of the control. The experiment was performed in triplicate, and three independent experiments were performed. The lowest concentration of propolis extracts that significantly increased cell proliferation was used in subsequent experiments.

### 2.9. Cell Migration Assay

The modified blind-well Boyden chamber migration assay was performed to evaluate the effect of the propolis extracts on HGF cell migration. The modified Boyden chemotaxis chamber (Neuro Probe, Gaithersburg, MD, USA) was used based on a chamber with two medium-filled compartments by modifying a previous method [27]. Briefly, collagen type I (Sigma-Aldrich) was applied to a polycarbonate membrane filter (13 mm diameter, 8.0 mm pore size, Whatman). The filter was placed above the lower chamber that contained serum-free DMEM with 0.1% bovine serum albumin (BSA, Sigma). HGFs (1 × 10^4^ cells) were resuspended in HEP (15.62 *μ*g/mL), EEP (40 *μ*g/mL), or AEP (400 *μ*g/mL) diluted in DMEM containing 0.1% BSA and seeded into the upper well of the chamber. The cell without propolis extract treatment was used as control. The cells were incubated for 5 h, and the filters were fixed and stained with crystal violet for 30 min. The migrated cells were counted by three investigators using a microscope at 400x magnification. The migrated cell counts were averaged from five randomly selected fields. Three chambers were used in each treatment. Three independent experiments were performed.

### 2.10. Wound Scratch Assay

The scratch assay was performed to test the effect of the propolis extracts on wound closure by HGFs as previously described [26]. HGFs were cultured in 10% FBS DMEM in 6-well plates (1 × 10^6^ cells/ well) for 24 h. When the cells were 80–90% confluence, the medium was replaced with serum-free DMEM to minimally maintain HGF growth. After 24 h, artificial wounds were created in the monolayers by making a linear scratch in the center of each well using a 200 *μ*L pipette tip. Any cellular debris created from scratch was removed by gently washing the wells with PBS. The HGFs were treated with HEP (15.62 *μ*g/mL), EEP (40 *μ*g/mL), or AEP (400 *μ*g/mL) for 24 h. Cells without propolis extract treatment were used as the control. The images of five randomly selected areas on each well were captured using a microscope camera (Nikon, Japan). A mark was placed on the back of each random area of each well as a reference point for subsequent imaging. The area measurements were calculated using Image J software (National Institutes of Health, Bethesda, MD, USA) by measuring the gap that was closed by the cells. The percent closure of the scratch width was calculated using the following equation:

(3) $$\begin{array}{c} \text{wound closure}\left(\%\right)=\left[\frac{A_{T0}-A_{T24}}{A_{T0}}\right]\times 100, \end{array}$$

where A_T0_ is the area of wound measured immediately after scratching and A_T24_ is the area of wound measured 24 h after scratching. Three independent experiments were performed.

### 2.11. Statistical Analysis

The data analyses were performed using GraphPad Prism 7.04 software (GraphPad Software, La Jolla, CA, USA). The data are expressed as means and standard error of the mean (SEM) as previously recommended [28]. The means of the data in multiple groups were compared using one-way ANOVA followed by Dunnett's or Tukey's post hoc test. *P* ≤ 0.05 was considered statistically significant.

## 3. Results

### 3.1. Extracted Yield and TLC Analysis of Propolis Samples

In this study, *n*-hexane, ethyl acetate, and distilled water were evaluated to determine their effects on the extraction yield of propolis. The results demonstrated a difference in the extraction yield using different solvents. Among the solvents tested, HEP resulted in the highest extraction yield (38.88%), followed by ethyl acetate (19.84%) and distilled water (1.42%) (Table 1). This indicated that the extraction efficiency is higher in low-polar solvents.

TLC was used to investigate the chemical profile of HEP, EEP, and AEP compared with that of the crude ethanol extract. Most of the spots on the TLC plates from the propolis extracts in the current study were detected in visible light, UV254 nm, UV366 nm, and visible light after staining with the anisaldehyde-sulfuric acid reagent. There were 21 spots using the *n*-hexane, ethyl acetate, and formic acid solvent systems (7 for crude ethanol extract, 6 for HEP, 6 for EEP, and 2 for AEP) (Figure 2(a)). The ethyl acetate : methanol : formic acid solvent system revealed 7 spots (1 for crude ethanol, 1 for HEP, 1 for EEP, and 4 for AEP) (Figure 2(b)). Therefore, the combination of nonpolar solvents was appropriate to separate HEP and EEP, whereas the combination of polar solvents was effective in separating AEP. The TLC chromatogram revealed the presence of 7 compounds with Rf values of 0.36–0.8 in crude ethanol extract. HEP contained 6 compounds with Rf values of 0.42–0.8, whereas 6 compounds with Rf values of 0.36–0.8 were found in EEP. AEP contained 4 compounds with Rf values of 0.17–0.79 (Table 2).

### 3.2. Chemical Analysis of the Propolis Extracts by GC-MS

The HEP, EEP, and AEP extracts were analyzed using GC-MS to determine their chemical composition. The 7 compounds that are commonly found in propolis, (1) m-coumaric acid, (2) ferulic acid, (3) caffeic acid, (4) galangin, (5) naringenin, (6) apigenin, and (7) quercetin, were used as standard compounds in our study. The chemical profiling of the standard compounds and the 3 propolis extracts is presented as chromatograms in Figure 3. The 7 standard compound peaks were distributed over various retention times (Rt): m-coumaric acid (Rt = 28.9), ferulic acid (Rt = 33.19), caffeic acid (Rt = 34.09), galangin (Rt = 43.79), naringenin (Rt = 45.54), apigenin (Rt = 48.94), and quercetin (Rt = 49.78) (Figure 3(a)). The data indicated that HEP, EEP, and AEP had different chemical compositions (Figure 3(b)–3(d)).

The chemical component in each propolis extract was identified based on the Wiley Registry® 10th Edition/NIST 2014 Mass Spectral Library. The compounds in each extract were reported when their mass spectral match score was higher than 70. Forty-four compounds met the criteria and were characterized as triterpenoids, tetraterpenoids, phenolics, flavonoids, alkaloids, sugars, and other compounds in HEP, EEP, and AEP (Table 3). The result revealed a high amount of triterpenoids (82.97%) in HEP. Phenolic compounds (65.15%) were identified as the most common components in EEP. However, triterpenoid and phenolic groups were not detected in AEP. Apigenin was identified as a flavonoid group in a very low amount (3.48%) in EEP, but not in HEP or AEP. Moreover, a high amount of sugar (84.55%) was identified as a major component in AEP but was not detected in HEP or EEP.

### 3.3. *In Vitro* Antioxidative Effect of Propolis Extracts

To evaluate the free radical scavenging activity in the propolis extracts, DPPH and FRAP assays were performed. The results demonstrated a similar pattern of antioxidant activity in the DPPH and FRAP assays (Figure 4). Quercetin (10 *μ*g/mL) was used as a positive control in the DPPH and FRAP assays. All propolis extracts exhibited antioxidant activity but significantly lower than that of quercetin (*P* < 0.05). However, the HEP and EEP exhibited significantly higher antioxidant activity than that of AEP in the DPPH assay (*P* < 0.05) (Figure 4(a)). The FRAP assay revealed that HEP had the highest antioxidant activity, followed by EEP and AEP (Figure 4(b)).

### 3.4. Proliferative Effect of Propolis Extracts on HGF

The 3 propolis extracts were evaluated for their proliferative effect on HGFs using an MTT assay. The propolis extracts demonstrated different effective concentration ranges. HEP exhibited a biphasic effect on cell proliferation with significantly increased cell proliferation at 15.62 and 31.25 *μ*g/mL compared with that of control (*P* < 0.05). In contrast, significantly inhibited cell proliferation was found when the concentration was increased to 250 *μ*g/mL (*P* < 0.05) (Figure 5(a)). EEP revealed a similar pattern of cell proliferation effect to that of the HEP, but at different concentrations. EEP significantly increased cell proliferation at 40 *μ*g/mL compared with that of control (*P* < 0.05); however, significantly inhibited cell proliferation was found when the concentration was increased to 320 *μ*g/mL (*P* < 0.05) (Figure 5(b)). AEP significantly increased HGF proliferation at a relatively high concentration (400 *μ*g/mL) compared with that of control (*P* < 0.05); however, there was no significant difference when the concentration was increased to 1,000 *μ*g/mL (*P* > 0.05) (Figure 5(c)). The minimum concentrations that significantly increased cell proliferation were used for the subsequent experiments. The selected concentrations were 15.62, 40, and 400 *μ*g/mL for HEP, EEP, and AEP, respectively.

### 3.5. Effect of Propolis Extracts on HGF Migration

The HGFs were treated with 15.62 *μ*g/mL HEP, 40 *μ*g/mL EEP, or 400 *μ*g/mL AEP, and cell migration was evaluated using a modified blind-well Boyden chamber migration assay. The migrating cells were stained with crystal violet after incubating with or without propolis extracts (Figure 6(a)). The migrating cells were counted using a light microscope at 400x magnification, and the mean migrating cells were calculated. The results indicated that cell migration significantly increased in HEP and EEP compared with that of control (*P* < 0.05) (Figure 6(b)). However, there was no significant difference in cell migration in AEP compared with that of control (*P* > 0.05).

### 3.6. Propolis Extracts Enhanced Wound Healing *In Vitro*

The scratch assay was employed to simultaneously evaluate the effect of the propolis extracts on HGF cell proliferation and migration. HGFs were treated with HEP, EEP, and AEP at their effective concentrations.  Figure 7(a) illustrates the wound closure with or without propolis extracts at the starting time (T0) and 24 h incubation (T24). The percentage of wound closure was measured and calculated using Image J software. The results indicated that the propolis extracts induced HGF wound healing activity by significantly increasing the percentage of wound closure compared with that of control (*P* < 0.05) (Figure 7(b)).

## 4. Discussion

The present study analyzed the phytochemical profile and the antioxidant activity of sequential hexane, ethyl acetate, and aqueous extracts of Thai propolis and determined their effects on human gingival fibroblast migration and proliferation. We found that the extraction yield of Thai propolis was the highest in the nonpolar solvent and gradually decreased with increasing polarity of the extract solvent. This suggests that the differential distribution of extracted compounds in the polar and nonpolar solvents was based on their polarity. Based on the polarity scale, water has the highest polarity of 9.0, and ethyl acetate has a medium polarity of 4.3, while hexane has the lowest polarity of 0.00 [29]. Thus, the composition and activity of the extracts will depend on the extraction method. More polar solvents will lead to better extraction of polar molecules, while nonpolar solvents will extract nonpolar molecules. Organic polar solvents result in a good extraction yield of both nonpolar and polar molecules [30, 31]. Our results demonstrated that *n*-hexane was the most effective method of raw propolis extraction to obtain the most chemically complex product. These results did not agree with the findings of the other studies that used ethanol extraction for processing raw propolis [32, 33].

The TLC of the crude ethanol extract, HEP, EEP, and AEP demonstrated that the resolution of the nonpolar eluent was greatest compared with the polar-mobile solvent. In addition, we found that the crude ethanol extract, HEP, and EEP had spots that reflected blue fluorescent in UV366 nm and became purple after staining with an anisaldehyde-sulfuric agent. Therefore, it is likely that most compounds in the crude ethanol, HEP, and EEP are terpenoids [19,34].

To date, numerous studies have been published regarding the chemical composition and biological effects of propolis. However, analysis of a large number of samples from different geographic regions has revealed that its chemical composition is highly variable and difficult to establish because it depends on several factors, including the vegetation and season at the collection site and the bee species. The main chemical groups present in propolis comprise phenolic compounds, such as esters, flavonoids, terpenes, aromatic aldehydes and alcohols, fatty acids, stilbenes, and *β*-steroids. Flavonoids have been reported to be the main compounds in propolis. Terpenoids, which represent only 10% of the content, are responsible for propolis' odor because they are volatile components in plants and contribute to their biological properties [35]. Surprisingly, Thai propolis had a very different flavonoid : terpenoid ratio compared with that of the other types of propolis [7, 36]. The GC-MS analysis in this study indicated that polyphenols and flavonoids were observed in low amounts in the propolis samples. Moreover, our standard compounds, m-coumaric acid, ferulic acid, caffeic acid, galangin, naringenin, apigenin, and quercetin, were not found in HEP, EEP, or AEP. In contrast, triterpenoids were markedly present in our samples, especially in HEP. We are the first to report that triterpenoids are the major compounds detected in Thai propolis from the *Tetragonula fuscobalteata* species. Our propolis chemical profile is similar to that of propolis from tropical areas that are enriched in triterpene. Triterpene-rich propolis was found in propolis samples from Malaysia [37], Yemen [38], Ethiopia [39], Bolivia [40], and Cameroon [41]. In contrast, propolis from temperate regions, such as France and Canada, contains mainly aromatic acids and their esters, flavonoids, and sugar derivatives with only traces of triterpenoids [42,43]. This confirms that the chemical composition of propolis varies by region depending on the local environment. Many studies on different samples have revealed that propolis' chemical composition is not consistent between regions because it is highly dependent on multiple factors, such as the environmental conditions at the site where the propolis resin is collected [41]. Our data suggest that propolis from Thailand is a promising new source of bioactive molecules.

The antioxidant activity of triterpenoid was observed in propolis from Cameroon [44], a medicinal fungus, *Sanghuangporus sanghuang* [45], and the stem bark of *Reissantia indica* [46]. It is possible that cycloartenol, *α*-amyrin, and *β*-amyrin that are classified as triterpenoids in the extract may have a synergistic effect on the antioxidant activity of HEP [47–49]. In contrast, the low antioxidant activity of EEP may be partly derived from phenolic compounds. Triterpenoids might not play a significant role in antioxidation in EEP because there were relatively high amounts of phenolic compounds compared with triterpenoids in this fraction. However, it should be noted that the amount of phenols and flavonoids in propolis might not always reflect their antioxidant capacity [50, 51].

The term antioxidant covers a wide range of different molecules; however, a common feature is their ability to readily donate electrons while remaining stable, thus acting as reducing agents and minimizing the damage caused by free radicals [52]. Antioxidants can be classified as primary or secondary. Primary antioxidants are free radical scavengers that inhibit or delay the initiation and/or propagation of free radicals by hydrogen atom transfer and single electron transfer. In contrast, secondary antioxidants do not convert free radicals into more stable products but act indirectly by decreasing the rate of oxidation by chelating prooxidant metals, replenishing hydrogen to primary antioxidants, absorbing ultraviolet radiation, or functioning as singlet oxygen quenchers [53]. Many antioxidant protocols have been devised to determine the antioxidant status of plants. Of particular interest are the ferric reducing antioxidant power assay (FRAP) using the single electron transfer reaction and DPPH using the hydrogen atom transfer reaction [54]. The DPPH results indicated that our propolis extracts acted as primary antioxidants through the donation of hydrogen.

The DPPH-free radical scavenging by antioxidants is due to their hydrogen-donating ability. Therefore, DPPH radicals are scavenged by antioxidants through the donation of hydrogen, forming reduced DPPH [55]. In the present study, the highest radical scavenging activity was observed in HEP and the lowest in AEP. The statistical analysis revealed a significant difference in radical scavenging activity between the three propolis extracts. The DPPH assay is often used to evaluate the ability of antioxidants to scavenge free radicals, which are known to be a major factor in biological damage caused by oxidative stress. This assay provides reliable information concerning the antioxidant ability of the tested compounds. DPPH radical formation involves a hydrogen atom transfer process [56, 57]. In this assay, the moderate antioxidant activity on DPPH radicals in HEP may be attributed to a direct role in trapping free radicals by donating hydrogen atoms.

The FRAP assay is based on the rapid reduction in ferric-tripyridyltriazine by antioxidants present in the samples forming ferrous-tripyridyltriazine, a blue-colored product [58]. In contrast to DPPH, the FRAP assay is the only assay that directly measures antioxidants (or reductants) in a sample compared with other assays that measure inhibition of free radicals. The values expressed from the FRAP assay represent the corresponding concentration of electron-donating antioxidants with the reduction of the ferric iron (Fe^3+^) to the ferrous ion (Fe^2+^) [59]. In our study, the strongest FRAP activity was exhibited by HEP and the lowest by AEP. We have shown that the FRAP and DPPH assays provide comparable results, which suggests that the reducing activity is a result of interaction between specific components. In this study, HEP was observed to have the highest antioxidation activity, which might be attributed to the nonpolar compounds, such as triterpenoids, in the extract. This hypothesis may be supported by the high amount of triterpenoids in HEP. Our results were consistent with previous studies [37, 41, 60]. However, our findings did not agree with other previous studies that demonstrated that polar solvents were better at extracting antioxidants from propolis and by extension improved the antioxidant properties compared with nonpolar solvents [15, 61]. There are multiple reports on the antioxidant effects of propolis [7, 62, 63]. The relationship between antioxidant activity and the chemical composition of propolis from different origins has been investigated by several groups [64–67]. These studies suggest that the high antioxidant activity of propolis is related to its high content of polyphenolic compounds, such as flavonoids [13, 60]. This suggests that different compositions in different propolis samples may exhibit some similar functions, such as antioxidant activity. Although HEP had a small amount of phenolic compounds, which are known as potential antioxidant agents [68], its activity might be mainly attributed to triterpenes in the extract [41].

The purpose of this study was to test the hypothesis that the antioxidant compounds in Thai propolis extracts stimulate HGF cell behaviors that increase wound healing in an *in vitro* model. Therefore, the effects of HEP, EEP, and AEP on HGF proliferation, migration, and *in vitro* wound healing were evaluated in the present study. Here, we demonstrated that Thai propolis extracts stimulated HGF proliferation and migration. HGF cells are known to play an essential role in wound healing. Cell migration is one of the most essential steps during the proliferative phase, which is responsible for wound closure [3]. HEP demonstrated the highest stimulation of HGF proliferation, followed by EEP and AEP. HGF migration was significantly increased in HEP and EEP, but not AEP. However, all three propolis extracts enhanced *in vitro* oral wound closure. This indicates that the propolis extracts, especially HEP and EEP, stimulate the proliferative phase of oral wound healing, especially oral fibroblast migration and proliferation. Our findings are in line with a previous study [11] that demonstrated that Malaysian and Brazilian red propolis stimulated human skin fibroblast proliferation, migration, and wound closure.

Wound healing requires a fine balance between the positive and deleterious effects of reactive oxygen species (ROS), a group of extremely potent molecules that are rate limiting in successful tissue regeneration. A balanced ROS response will debride and disinfect a tissue and stimulate healthy tissue turnover, suppressed ROS will result in infection, and increased ROS will destroy otherwise healthy stromal tissue [69]. The homeostatic control of cellular ROS levels (redox state) is modulated by proteins known as antioxidants. Antioxidants are proteins that reduce the deleterious effects of ROS by donating their own electrons, thus preventing them from capturing electrons from other important molecules, such as DNA, proteins, and lipids [4].

Antioxidants are proposed to control wound oxidative stress and thereby accelerate skin and oral wound healing [70, 71]. Potent antioxidants play an important role in periodontal wound healing because chronic inflammation, excessive reactive oxygen species (ROS) production, and oxidative stress are key contributors to the host connective tissue damage associated with periodontal disease pathogenesis [72–74]. Many facets of wound healing under redox control require a delicate balance between oxidative stress and antioxidants. Although the normal physiology of wound healing depends on low levels of reactive oxygen species and oxidative stress, overexposure to oxidative stress leads to impaired wound healing. Our findings demonstrated that the different antioxidant activities of the propolis extracts had similar effects on cell proliferation, cell migration, and *in vitro* wound closure. Therefore, our results confirm those of previous studies that reported that antioxidant compounds in the propolis extract play an important role in wound healing [12, 13].

Two systematic reviews revealed that triterpenes induce wound healing [75, 76]. These compounds increase the success rate of wound healing, the rate of epithelialization, and collagen deposition in tissues. However, further investigation is required to clarify the molecule targets through which triterpenoids mediate healing effects. In this study, the GC-MS chromatograms revealed a high content of triterpenoids (82.97%) in HEP that may contribute to the potential increased oral wound healing effect of Thai propolis.

The results of this study have some implications for the clinical use of propolis extracts in oral wound healing. However, wound healing has various stages and is facilitated by antioxidant, antimicrobial, and anti-inflammatory activities. Therefore, further investigations need to be performed on the effect of this propolis on the other processes of wound healing. In addition, experiments should be performed using different cell types involved in oral wound healing.

This study has some limitations that need to be considered when interpreting the results. The present study was performed using an *in vitro* oral wound healing model. This model may not fully reflect the overall oral wound healing processes. Therefore, this study should be repeated using an animal model. Another limitation is that this study did not identify the exact bioactive components that regulate our observed HGF behaviors. To overcome these limitations, future studies are necessary to identify the bioactive components involved in oral wound healing activation from Thai propolis.

However, in line with the previous reports, our data support that propolis at a defined concentration is cytocompatible and, thus, may be used as an adjuvant therapeutic supplement that has the potential to enhance oral wound healing.

## 5. Conclusion

Within the scope of this study, we have demonstrated that the *n*-hexane extract and ethyl acetate extracts of Thai propolis enhance the proliferative phase of oral wound healing. The extracts also stimulate the proliferation of human gingival fibroblasts. However, the effect of the aqueous extract of propolis on antioxidation and cell migration was scant compared with the *n*-hexane and ethyl acetate extracts. Furthermore, the effect of bioactive compounds identified in our propolis on *in vivo* oral would healing is needed to be addressed.

## Figures and Tables

**Figure 1:** Flowchart of the propolis extraction and solvent partitions. HEP, EEP, and AEP were obtained. The dry weight of each sample was indicated.

**Figure 2:** TLC analysis of the propolis samples. TLC profiling of the propolis extracts using (a) hexane/ethyl acetate/formic acid (30 : 70 : 1) and (b) ethyl acetate/methanol/formic acid (50 : 50 : 1) solvents. The TLC analysis was visualized under UV254 nm, UV366 nm, and an anisaldehyde-sulfuric acid agent compared with that of natural light. Samples no.1, 2, 3, and 4 represent the crude extract, hexane, ethyl acetate, and aqueous extracts, respectively.

**Figure 3:** GC-MS chromatograms of the standard compounds and propolis extracts. The chromatograms were plotted between total ion count and acquisition time of standards and the propolis fractions. (a) Chromatogram demonstrates the peaks of the 7 standard compounds: (1) m-coumaric acid, (2) ferulic acid, (3) caffeic acid, (4) galangin, (5) naringenin, (6) apigenin, and (7) quercetin. The chemical profiles of (b) HEP, (c) EEP, and (d) AEP are shown.

**Figure 4:** *In vitro* antioxidative effect of propolis extracts. (a) Free radical scavenging activity in each propolis extract (500 *μ*g/ml) was evaluated by DPPH assay (*n = 3).* (b) Ferric radical scavenging activity in each propolis extract (500 *μ*g/ml) was evaluated by FRAP assay *(n* = 3). Quercetin (10 *μ*g/mL) was used as the positive control. Bars represent the mean ± SEM of the percentage of free radical scavenging. ^*∗*^*P* < 0.05 versus the quercetin, ^#^*P* < 0.05 versus HEP, ^$^*P* < 0.05 versus EEP.

**Figure 5:** Proliferative effect of propolis extracts on HGFs. The cells were treated with 3 propolis extracts at various concentrations for 72 h. Cells in media without propolis extract were used as control. MTT assay was used to evaluate the cell proliferation effect of (a) HEP (15.62, 31.25, 62.5, 125, and 250 *μ*g/mL), (b) EEP (20, 40, 80, 160, and 320 *μ*g/mL), and (c) AEP (200, 400, 600, 800, and 1000 *μ*g/mL) (n = 3). Bars represent the mean ± SEM of cell proliferation (% of control). ^*∗*^*P* < 0.05 versus the control group.

**Figure 6:** Effect of propolis extracts on HGF migration. The effective doses of propolis extracts, HEP (15.62 *μ*g/mL), EEP (40 *μ*g/mL), and AEP (400 *μ*g/mL), were used to treat the HGFs for 5 h in blind-well Boyden chambers. Cells in media without propolis extract were used as control. (a) The migrating cells were stained with crystal violet for 30 min. Scale bar = 100 *μ*m. The migrated cells were counted under a light microscope in 5 random fields at 400x magnification. (b) The average migrated cell was calculated for each group (n = 3). Bars represent mean ± SEM of migrating cell no./field. ^*∗*^*P* < 0.05 versus the control group.

**Figure 7:** Propolis extracts enhanced wound healing *in vitro*. The effective doses of propolis extracts, HEP (15.62 *μ*g/mL), EEP (40 *μ*g/mL), and AEP (400 *μ*g/mL), were used to treat the HGFs for 24 h. The cells in media without propolis extract were used as control. (a) Scratch assay results. The wound closure pictures were taken at the initial time (T0) and after 24 h incubation (T24). Scale bar = 100 *μ*m. (b) The wound distance in each group was measured at each time point and calculated as the percentage of wound closure using Image J software (n = 3). Bars represent the mean ± SEM of the percentage of wound closure. ^*∗*^*P* < 0.05 versus the control group.

**Table 1:** The HEP, EEP, and AEP extract yields.

Extract results	Extracts		
	HEP	EEP	AEP
Extract yield (g)	63.37	32.34	2.33
Percentage yield (% W/W)	38.88	19.84	1.42

**Table 2:** Rf values of the propolis crude ethanol, HEP, EAP, and AEP.

Spots	Crude ethanol extract^*∗*^	Spots	HEP^*∗*^	Spots	EEP^*∗*^	Spots	AEP^#^
A	0.80	A	0.80	A	0.72	A	0.79
B	0.72	B	0.72	B	0.65	B	0.68
C	0.65	C	0.65	C	0.59	C	0.45
D	0.59	D	0.59	D	0.45	D	0.17
E	0.45	E	0.45	E	0.42		
F	0.42	F	0.42	F	0.36		
G	0.36						

^*∗*^Mobile phase: *n*-hexane, ethyl acetate, and formic acid (30 : 70 : 1). ^#^Mobile phase: ethyl acetate, methanol, and formic acid (50 : 50 : 1).

**Table 3:** Characterization of the compounds in the propolis extracts by GC-MS.

Retention time (min)	Compounds	Formula	Composition in propolis extracts (% peak area)		
			HEP	EEP	AEP
	Triterpenoid				
50.81	23-(Phenylsulfanyl) lanosta-8,24-dien-3-ol	C_36_H_54_OS	2.26	—	—
51.60	*β*-Amyrin	C_30_H_50_O	9.70	6.63	—
51.74	*β*-Amyrone	C_30_H_48_O	6.56	—	—
51.80	Lupenone	C_30_H_48_O	1.18	—	—
51.91	13,27-Cycloursan-3-one (Phyllanthone)	C_30_H_48_O	9.66	—	—
52.14	*α*-Amyrin	C_30_H_50_O	9.98	6.15	—
52.23	Lupeol	C_30_H_50_O	4.27	2.91	—
52.49	Cycloartenol	C_30_H_50_O	29.24	13.27	—
52.81	Toosendanin (Chuanliansu)	C_30_H_38_O_11_	2.38	—	—
53.04	24-Methylenecycloartanol acetate	C_33_H_54_O_2_	5.99	—	—
53.55	Betulinaldehyde	C_30_H_48_O_2_	1.75	—	—
	Tetraterpenoid				
52.94	Dimethoxylycopene	C_42_H_64_O_2_	1.85	—	—
	Phenolic				
22.24	3-Hydroxybenzoic acid (m-Salicylic acid)	C_7_H_6_O_3_	—	—	0.42
27.95	3,5-Dihydroxybenzoic acid (*α*-resorcylic acid)	C_7_H_6_O_4_	—	—	1.19
42.53	3-(10-Heptadecenyl)phenol (Cardanol C17:1)	C_23_H_38_O	1.66	2.24	—
42.64	2',5'-Dimethoxyoctadecanophenone	C_26_H_44_O_3_	0.86	—	—
42.80	5-(8Z-Pentadecenyl)resorcinol (Bilobol C15:1)	C_21_H_34_O_2_	—	3.64	—
44.97	Hydroginkgolic acid (Anacardic acid C15:0)	C_22_H_36_O_3_	0.76	—	—
45.45	3-(nonadec-12-en-1-yl)phenol (Cardanol C19:1)	C_25_H_42_O	5.67	—	—
45.22	(Z)-5-(heptadec-10-en-1-yl)resorcinol (Bilobol C17:1)	C_23_H_38_O_2_	3.17	40.44	—
47.57	2-[(Z)-heptadec-10-enyl]-6-hydroxybenzoic acid (Ginkgolic acid C17:1)	C_24_H_38_O_3_	3.06	7.96	—
50.11	6-[12(Z)-Nonadecenyl]salicylic acid (Ginkgolic acid C19:1)	C_26_H_42_O_3_	—	10.87	—
	Flavonoid				
51.72	Apigenin, 7-O-sophoroside	C_27_H_30_O_15_	—	3.48	—
	Alkaloid				
29.17	Quininic acid	C_11_H_9_NO_3_	—	—	3.00
	Sugar				
24.52	D-Ribose	C_5_H_10_O_5_	—	—	0.48
28.22	D-(+)-Talofuranose; Talose's isomer	C_6_H_12_O_6_	—	—	1.62
28.37	Methyl galactoside	C_7_H_14_O_6_	—	—	1.35
29.74	*α*-Methylglucoside	C_7_H_14_O_6_	—	—	0.29
30.04	Talose	C_6_H_12_O_6_	—	—	0.76
44.22	D-(-)-Fructofuranose; Fructose's isomer	C_6_H_12_O_6_	—	—	3.40
44.83	3-*α*-Mannobiose; 3-O-alpha-D-Mannopyranosyl-D-mannopyranose	C_12_H_22_O_11_	—	—	0.67
54.97	D-(+)-Turanose	C_12_H_22_O_11_	—	—	0.29
	Sugar acid				
22.16	L-Threonic acid	C_4_H_8_O_5_	—	—	0.68
23.99	Arabinonic acid, *γ*-lactone	C_5_H_8_O_5_	—	—	0.42
27.55	Ribonic acid	C_5_H_10_O_6_	—	—	1.92
29.81	Gulonic acid, *γ*-lactone	C_6_H_10_O_6_	—	—	1.52
31.91	Galactonic acid	C_6_H_12_O_7_	—	—	3.50
31.98	D-Gluconic acid	C_6_H_12_O_7_	—	—	1.43
37.08	Glyceryl glucoside	C_9_H_18_O_8_	—	—	1.42
	Sugar alcohol				
8.55	2,3-Butanediol	C_4_H_10_O_2_	—	—	0.29
15.27	Glycerol	C_3_H_8_O_3_	—	—	23.29
21.16	L-Threitol	C_4_H_10_O_4_	—	—	1.24
21.40	Erythritol	C_4_H_10_O_4_	—	—	20.06
25.97	L-(-)-Arabitol	C_5_H_12_O_5_	—	—	0.64
26.27	Xylitol	C_5_H_12_O_5_	—	—	4.27
26.94	1,5-Anhydrohexitol; Polygalitol	C_6_H_12_O_5_	—	—	0.31
28.49	3-Deoxyhexitol	C_6_H_14_O_5_	—	—	1.26
30.61	D-Mannitol	C_6_H_14_O_6_	—	—	3.82
30.77	D-Sorbitol	C_6_H_14_O_6_	—	—	5.33
30.85	Dulcitol; Galactitol	C_6_H_14_O_6_	—	—	2.00
33.51	Myo-Inositol	C_6_H_12_O_6_	—	—	1.51
46.64	Maltitol	C_12_H_24_O_11_	—	—	0.78
	Others				
9.19	D-(-)-Lactic acid	C_3_H_6_O_3_	—	—	6.82
16.02	Butanedioic acid; Succinic acid	C_4_H_6_O_4_	—	—	1.25
18.59	2-Methylglutaric acid	C_6_H_10_O_4_	—	2.40	—
28.27	Isocitric acid	C_6_H_8_O_7_	—	—	0.29
29.61	Nonadecanoic acid; Nonadecylic acid	CH_3_(CH_2_)_17_˗COOH	—	—	2.50

## Data Availability

The datasets used and/or analyzed during the current study are available from the corresponding author upon request.
